The article "Research on User Experience of Sports Smart Bracelet Based on Fuzzy Comprehensive Appraisal and SSA-BP Neural Network" was retracted in 2023. Reasons: suspected computer-generated content; unreliable results or conclusions; concerns about the data; concerns about the results or conclusions.

# Research on User Experience of Sports Smart Bracelet Based on Fuzzy Comprehensive Appraisal and SSA-BP Neural Network

**DOI:** 10.1155/2022/5597662

**Published:** 2022-01-05

**Authors:** Xichun Luo, Honghao Zhao, Yan Chen

**Affiliations:** ^1^School of Intelligent Manufacturing, Dongguan City College, Dongguan, Guangdong 523000, China; ^2^Department of Decision Sciences, School of Business, Macau University of Science and Technology, Taipa, Macao 999078, China; ^3^School of Creative Design, Dongguan City College, Dongguan, Guangdong 523000, China

## Abstract

Due to the marked increase in the prevalence of overweight and obesity worldwide and an environment leading to a series of chronic diseases, physical exercise is an important way to prevent chronic diseases. Additionally, a good exercise smart bracelet can bring convenience to physical exercise. Quick and accurate evaluation of smart sports bracelets has become a hot topic and draws attention from both academic researchers and public society. In the literature, the analytic hierarchy process (AHP) and entropy weight method (EWM) were used to obtain the weights from both subjective and objective perspectives, which were integrated by the comprehensive weighting method, and furthermore the performance of sports smart bracelet was evaluated through fuzzy comprehensive evaluation. Also, to avoid complex weight calculations caused by the comprehensive weighting method, machine learning methods are used to model the structure and contribute to the comprehensive evaluation process. However, few studies have investigated all previous elements in the comprehensive evaluation process. In this study, we consider all previous parts when evaluating smart sports bracelets. In particular, we use the sparrow search algorithm (SSA) to optimize the backpropagation (BP) neural network for constructing the comprehensive score prediction model of the sports smart bracelet. Results show that the sparrow search algorithm-optimized backpropagation (SSA-BP) neural network model has good predictive ability and can quickly obtain evaluation results on the premise of effectively ensuring the accuracy of the evaluation results.

## 1. Introduction

In recent years, the frequency of overweight and obesity has increased significantly worldwide [1]. In China, the prevalence of overweight and that of obesity have risen from 37.4% and 8.6% to 41.2% and 12.9%, respectively, and have become a major public health concern [2]. Studies have shown that overweight and obesity induce chronic diseases such as hypertension, diabetes, and cardiovascular diseases and can lead to shortened life expectancy [3, 4]. Regular exercise is helpful to prevent chronic diseases, improve quality of life, and promote physical and mental health [5, 6].

Therefore, participation in sports and appropriate physical activities plays an important role in preventing chronic disease [7]. According to a number of studies, AI sports equipment with exercise programs may increase positivity [8, 9]. Among them, smart sports bracelets are a commonly used intelligent wearable device in sports today [10, 11]. By collecting data and browsing health records, sports smart bracelets can monitor physiological data during exercise [12].

Therefore, before developing new sports smart wristbands, user experience research on existing products can improve the practicability of product development and thus play a role in the healthy life of users. In the academic world, some scholars have performed systematic evaluations of products through various evaluation methods, providing a theoretical basis for designers to improve design and scheme decisions. Zheng et al. [13] established a comprehensive model of user satisfaction of public fitness equipment with the use of the fuzzy analytic hierarchy process, understood the satisfaction of users in the real experience process, and proposed the direction and design of optimization and improvement based on the importance of user experience elements expressed in the feedback of device satisfaction according to the importance-performance analysis (IPA) quadrant diagram. Xia et al. [14] applied a combination of analytic hierarchy process (AHP) and a fuzzy comprehensive evaluation method to evaluate health apps for the elderly and proposed that more considerations should be given to the physical and psychological factors of the elderly when designing health application procedures for the elderly. Chang et al. [15] established a quantitative evaluation model for the design of sweepers by combining AHP and fuzzy comprehensive evaluation. This scored three modeling design schemes of small electric four-wheel sweepers and identified the best design scheme, which provided a reference for the modeling design and evaluation of sweeper and similar products. Li et al. [16] considered three aspects of product pricing, hardware configuration, and software configuration; established the product optimization evaluation model of Kindle e-reader using entropy TOPSIS (Technique for Order Preference by Similarity to an Ideal Solution) method; and proposed decision-making opinions for the optimization and development of Kindle electronic creative products. Hayat et al. [17] proposed that when developing new products, customer preferences should be determined based on customer requirements for acceptability and satisfaction levels; Shannon entropy should be used to weight these preferences; and TOPSIS should be used to obtain a comprehensive evaluation of the product. Results show that this approach is reasonable and can provide a realistic and flexible framework for two or more clients to choose design solutions.

In addition, scholars' comprehensive evaluation of other fields also has lent credibility to this study. Ma et al. [18] evaluated the development status of new energy vehicles in China, Japan, Germany, and the United States with a series of indicators, such as technological innovation, market development, and infrastructure construction level, using the AHP and entropy weight method (EWM) to combine subjective and objective factors. Studies show that Germany has the strongest comprehensive development status, and other countries lead in different indicators. Zhang et al. [19] constructed an evaluation model of water resource value in Wuhan based on the AHP, the EWM, and the fuzzy comprehensive evaluation method, providing a decision-making basis for the government to reasonably determine water prices, evaluate local natural resource assets, and compile natural resource balance sheets.

Table 1 shows that Zheng et al., [13] Xia et al. [14], and Chang et al. [15] only use the AHP to directly combine with fuzzy comprehensive evaluation. AHP is subjective when determining product design elements. Thus, the weight of each design element is not accurate and scientific, making the choice of the best design scheme inaccurate. However, Li et al. [16] and Hayat et al. [17] only use the EWM, which primarily mines information from index data and is easily divorced from the real situation of evaluation. Ma et al., Zhang et al. [18], and Ma et al. [19], through the AHP and EWM, combined subjective and objective methods to determine the weight to obtain a more reliable comprehensive weight; however, their evaluation objects were not product design. In the field of comprehensive evaluation, few scholars have applied subjective and objective evaluation methods to product design decision-making. This study aims to fill this gap.

In addition, to avoid complex weight calculations, after establishing the fuzzy comprehensive evaluation system, this study directly predicts the comprehensive score using the personal score by constructing the prediction model of data mining. In the work of Chen et al. [20], during the COVID-19 pandemic, a backpropagation (BP) neural network model was used to predict users' satisfaction with online teaching, and the prediction accuracy reached 77.5%. Kalinic et al. [21] used a BP neural network to predict mobile commerce consumer satisfaction and found that neural networks have higher predictive abilities than linear models. Liu et al. [22] optimized the extreme learning machine (ELM) through sparrow search algorithm (SSA) to predict short-term wind power production. Simulation results show that the proposed SSA-ELM model has a high prediction accuracy and a strong generalizability, which provides decision support for wind power prediction and stable operation of power grid security.

Combining these studies in the field of satisfaction prediction, the BP neural network achieves good predictions, and the SSA intelligent optimization algorithm can be used to optimize the machine learning model and improve the prediction accuracy of the model. Therefore, this study uses a BP neural network to predict the comprehensive score of the exercise intelligent bracelet, optimizes it based on SSA, and obtains a comprehensive evaluation model of the exercise intelligent bracelet based on SSA-BP.

The contributions of this study are as follows:

1. A thorough comprehensive evaluation process is investigated to evaluate smart sports bracelets, which includes using the AHP, EWM, and fuzzy comprehensive evaluation models for comprehensive score construction and the implementation of the SSA-BP neural network for comprehensive score prediction.
2. AHP and EWM are used to determine weights from both subjective and objective perspectives from experts and users. These weights are combined with the comprehensive weighting method, and the fuzzy comprehensive evaluation method is used to evaluate the sports smart bracelet to improve the reliability of product evaluation and provide a decision basis for designers.
3. The SSA optimized BP neural network is used to comprehensively evaluate the sports smart bracelet to avoid cumbersome weight calculations and quickly obtain the evaluation results to ensure the accuracy of the evaluation results.

Finally, the remainder of this paper is structured as follows: Section 2 selects the evaluation indicator of the sports smart bracelet; Section 3 constructs the fuzzy comprehensive evaluation model based on the AHP and EWM; Section 4 uses the SSA-BP neural network to construct the comprehensive score prediction model; Section 5 verifies the feasibility of the proposed method using a practical case of sports smart bracelets; and Section 6 draws conclusions and recommends future research.

## 2. Evaluation Indicators of Sports Smart Bracelets

First, based on the results of existing evaluation methods for product design schemes and the characteristics of the smart sports bracelets, we preliminarily identified important evaluation indicators: size, interface design, clear interface, heart rate detection, motion function, and material elasticity [23]. Second, 10 sports smart bracelet users were selected for in-depth research, and the indicators in the model were added or deleted according to users' satisfaction perception. Finally, an in-depth interview was conducted with three industrial design experts; open questions were set on the rationality and integrity of the model indicators; and indicators were modified and improved according to the experts' opinions. These amendments were as follows:

1. Integration of indicator elements: integrate similar concepts, such as the appearance of the features of the “shell,” “interface” into the “size,” “easy to use interface navigation,” “reasonable interface design,” “clear interface,” and other indicators into the “touch interface”
2. Deletion of indicator elements: in the process of user interviews, some indicators were not mentioned, or the concept of fuzzy indicators was deleted, including “elasticity,” “skin affinity,” “multiple selection,” and other indicators in the material
3. Supplement of indicator elements: according to the user's description of the added value of the product, “product performance” is added

Finally, 16 evaluation indicators were used and divided into five first-level indicators: appearance characteristics, interactivity, functionality, material, and product characteristics. The evaluation indicator classification of sports smart bracelets is shown in Figure 1.

## 3. Comprehensive Evaluation Model of Sports Smart Bracelets

### 3.1. Construction of Evaluation Matrix

An evaluation factor set and comment set were developed. Factor set S was divided into *k* subsets according to the type of indicator attribute and was denoted as *S*={*S*_1_, *S*_2_,…, *S*_*k*_}, and the evaluation set P composed of different evaluation grades was denoted as *P*={*P*_1_, *P*_2_,…, *P*_*k*_}. The evaluation matrix *t* was used to represent the corresponding fuzzy membership degree of each indicator element, and the relation matrix of fuzzy membership degree was established as follows:

(1) $$\begin{array}{c} T=\left[\begin{array}{cccc} t_{11} & t_{12} & \ldots & t_{1n}\\ t_{21} & t_{22} & \ldots & t_{2n}\\ \vdots & \vdots & \; & \vdots \\ t_{m1} & t_{m2} & \ldots & t_{mn} \end{array}\right]\left(0\leq t_{ij}\leq 1\right), \end{array}$$

where *T* is the fuzzy evaluation relation matrix of all indicator dimensions; *t*_*ij*_ is the element in the *i*th row and *j*th column; and the row and column represent the indicator and comment level, respectively.

### 3.2. Determination of the Weight of Evaluation Indicators

In this study, the subjective AHP was first used to determine the weight, and then the objective EWM was used to determine the weight, and then the comprehensive weighting method was used to combine the two. The comprehensive weight was then determined.

#### 3.2.1. Analytic Hierarchy Process

The AHP was proposed by Saaty, an American operational research expert, in 1970 and has been widely applied in the field of decision-making [24–26]. In this study, the scale method of 1–9 in the AHP [27] is used to compare each evaluation indicator in the evaluation system in pairs to build a judgment matrix and calculate the corresponding weights of each first-level indicator and second-level indicator.

First, the judgment matrix is constructed based on the opinions of experts on each evaluation as follows:

(2) $$\begin{array}{c} D=\left[\begin{array}{cccc} d_{11} & d_{12} & \ldots & d_{mm}\\ d_{21} & d_{22} & \ldots & d_{mm}\\ \vdots & \vdots & \; & \vdots \\ d_{m1} & d_{m2} & \ldots & d_{mm} \end{array}\right]\left(0\leq d_{ij}\leq 1\right). \end{array}$$

In this study, the commonly used geometric average method is used, and its specific steps are as follows:

(1) Normalize each value in the judgment matrix *d* by column to obtain *g*_*ij*_:
  (3) $$\begin{array}{c} g_{ij}=\frac{d_{ij}}{\sum_{i=1}^{m}d_{ij}}. \end{array}$$
(2) Add the normalized values in rows to obtain *a*_*i*_:
  (4) $$\begin{array}{c} a_{i}=\sum_{j=1}^{m}g_{ij},\;j=1,2,\cdots ,m. \end{array}$$
(3) Normalize obtained *a*_*i*_ to obtain the relative weight *α*_*i*_:
  (5) $$\begin{array}{c} \alpha_{i}=\frac{a_{i}}{\sum_{i=1}^{m}a_{i}}. \end{array}$$

According to the requirements of the AHP, to ensure consistent thinking and the compatibility of the judgment matrix of the evaluators in the evaluation process, it is necessary to conduct a consistency test after solving the judgment matrix and weight of each element. CI is used to represent the consistency indicator of the judgment matrix:

(6) $$\begin{array}{c} \text{CI}=\frac{\lambda_{\max}-m}{m-1}, \end{array}$$

(7) $$\begin{array}{c} \text{CR}=\frac{\text{CI}}{\text{RI}}. \end{array}$$

RI is the random consistency index, as shown in Table 2. *λ*_max_ is the maximum characteristic quantity of the judgment matrix. *m* is the number of factors. If CR < 0.1, the judgment matrix meets the consistency requirement. Once CR ≥ 0.1, the judgment matrix needs to be modified until the consistency is reached.

#### 3.2.2. Entropy Weight Method

The EWM is widely used in the field of economic management and decision control [28, 29], and weight is determined by the size of the information of each evaluation indicator. When the information of the indicator directly changes markedly, the smaller the entropy value is, the greater the entropy weight is, indicating that the indicator is more important in the evaluation system.

Based on the evaluation matrix of equation (1), the steps of EWM are as follows:

(1) Conduct dimensionless processing of the original data to eliminate the influence of physical quantities:
  (8) $$\begin{array}{c} t_{ij}^{\prime }=\frac{t_{ij}-t_{ij\min}}{t_{ij\max}-t_{ij\min}}. \end{array}$$
(2) Calculate the *j*th grade, the proportion, or contribution of the *i*th evaluation indicator:
  (9) $$\begin{array}{c} p_{ij}=\frac{t_{ij}^{\prime }}{\sum_{j=1}^{n}t_{ij}^{\prime }}. \end{array}$$
(3) Calculate the entropy value of the *j*th evaluation indicator:
  (10) $$\begin{array}{c} e_{i}=-\frac{1}{\ln\;m}\sum_{j=1}^{n}p_{ij}\ln\left(p_{ij}\right),\;0\leq e_{i}\leq 1. \end{array}$$
(4) Calculation of difference coefficient is as follows:
  (11) $$\begin{array}{c} g_{i}=1-e_{i}. \end{array}$$
(5) Determine the weight of evaluation indicators *β*_*i*_:
  (12) $$\begin{array}{c} \beta_{i}=\frac{g_{i}}{\sum_{i=1}^{m}g_{i}},\;i=1,2,3,\cdots ,m. \end{array}$$

#### 3.2.3. Comprehensive Weighting Method

AHP primarily determines the weights based on the experience and knowledge of experts. Although AHP can combine the real evaluations, it is influenced by the personal preference of experts. The EMW primarily mines information from indicator data but is easily divorced from reality. Therefore, the comprehensive weighting method is used in this study to combine the subjective weight related to the experience of experts in related fields with the objective weight of information which describe indicators to jointly determine the comprehensive weight of evaluation indicators. The relevant formula is as follows:

(13) $$\begin{array}{c} w_{i}=\frac{\alpha_{i}\beta_{i}}{\sum_{i=1}^{m}\alpha_{i}\beta_{i}},\;i=1,2,3,\cdots ,m. \end{array}$$

### 3.3. Fuzzy Comprehensive Evaluation

To obtain the overall evaluation results of the sports smart bracelet, a multilevel fuzzy comprehensive evaluation model should be used to solve the problem; thus, the evaluation matrix of each indicator should be established to solve the second-level indicator evaluation, and then the second-level indicator evaluation matrix should be established to solve the evaluation results of the first-level indicators. We thus first set up the comment set and the factor set, establish the evaluation matrix from the second-level indicators, determine the membership degree of each comment in the comment set for each indicator in the factor set, and normalize the process. The evaluation vector *R*=(*r*_1_, *r*_2_, ⋯, *r*_*n*_) is composed of various factors including evaluation matrix *T*=(*t*_*ij*_)_*m*×*n*_ and the weight vector obtained by the comprehensive weighting method through fuzzy evaluation calculation, and the results are as follows:

(14) $$\begin{array}{c} R=W^{T}T={\left[\begin{array}{c} w_{1}\\ w_{2}\\ \vdots \\ w_{m} \end{array}\right]}^{T}\left[\begin{array}{cccc} t_{11} & t_{12} & \ldots & t_{1n}\\ t_{21} & t_{22} & \ldots & t_{2n}\\ \vdots & \vdots & \; & \vdots \\ t_{m1} & t_{m2} & \ldots & t_{mn} \end{array}\right]=\left(r_{1},r_{2},\cdots ,r_{n}\right), \end{array}$$

where *W*=(*w*_1_, *w*_2_, ⋯,*w*_*m*_)^*T*^ is the weight of all levels of indicators.

## 4. SSA-BP Neural Network

### 4.1. Sparrow Search Algorithm

The sparrow search algorithm is a novel swarm optimization approach proposed by Xue and Shen [30] which was inspired by the group wisdom, foraging, and anti-predation behaviors of sparrows. This algorithm is implemented by idealizing the behavior of the sparrows and formulating corresponding rules.

We assume that *n* sparrows exist in a *D*-dimensional space. The location of the *i*th sparrow in this *D*-dimensional space is denoted as *X*_*i*_={*x*_*i*1_, *x*_*i*2_,…, *x*_*i*  *d*_}, and its fitness values are given by *F*_*x*_*j*__=*f*({*x*_*i*1_, *x*_*i*2_,…, *x*_*i*  *d*_}). In each iteration, the sparrows with the higher energy act as the producers, and the remaining sparrows are chosen as the scroungers. In addition, 10% to 20% of the total sparrows that are aware of the danger act as the safeguard for generating alarms, and their locations are randomly generated in the population.

The location updating for producer is given by

(15) $$\begin{array}{c} X_{i,j}^{t+1}=\left\{\begin{array}{cc} X_{i,j}^{t+1}\times \;\exp\left(\frac{-i}{\alpha \times iter_{\max}}\right)\text{,} & \text{if }R^{2}<ST,\\ X_{i,j}^{t}+Q\times L, & \text{if }R^{2}\geq ST, \end{array}\right) \end{array}$$

where *t* is the current number of iterations and *j*={1,2, ⋯, *d*} is the number of dimensions. Also, *α* ∈ (0,1] is a random number, *iter*_max_ is the maximum number of iterations, *X*_*i*,*j*_^*t*^ is the location of the *i*th sparrow in the *j*th dimension at iteration *t*, *R*^2^ ∈ [0,1] is the alarm value, and *ST* ∈ [0.5, 1.0] is the safety threshold. The random number *Q* follows a standard normal distribution, and *L* is a 1 × *d* matrix with elements equal to 1.

In particular, *R*^2^ < *ST* indicates that no predators are present, and the producer enters the wide search mode. If *R*^2^ ≥ *ST*, then some sparrows have discovered a predator, and all sparrows must quickly fly to other safe areas.

Apart from the producers, the remaining sparrows act as scroungers, and their updated location is given by

(16) $$\begin{array}{c} X_{i,j}^{t+1}=\left\{\begin{array}{cc} Q\times \;\exp\left(\frac{X_{\text{worst}}^{t}-X_{i,j}^{t}}{i^{2}}\right),\; & \text{if }i>n/2,\\ X_{P}^{t+1}+\left|X_{i,j}^{t}-X_{P}^{t+1}\right|\times A^{+}\times L, & \text{otherwise,} \end{array}\right) \end{array}$$

where *X*_worst_^*t*^ is the current global worst location and *X*_*P*_^*t*+1^ is the optimal position occupied by the producer at iteration *t*+1. Also, *A*^+^=*A*^*T*^(*AA*^*T*^)^−1^, where A is a 1 × *d* matrix with elements that are randomly assigned 1 or −1, and *n* is the number of sparrows.

The location for sparrows that are aware of the danger is given by

(17) $$\begin{array}{c} X_{i,j}^{t+1}=\left\{\begin{array}{cc} X_{\text{best}}^{t}+\beta \times \left|X_{i,j}^{t}-X_{\text{best}}^{t}\right|\text{, } & \text{if }f_{i}>f_{g},\\ X_{i,j}^{t}+K\times \left(\frac{\left|X_{i,j}^{t}-X_{\text{worst}}^{t}\right|}{\left(f_{i}-f_{w}\right)+\varepsilon }\right), & \text{if }f_{i}=f_{g}, \end{array}\right) \end{array}$$

where *X*_best_^*t*^ is the current global optimal location; *β* is the step size control parameter and is a normal distribution of random numbers with a mean value of 0 and a variance of 1; and *K* ∈ [−1,1] is a random number and indicates the direction in which the sparrow moves and is also the step size control coefficient. Also, *ε* is the smallest constant to avoid zero-division error, *f*_*i*_ is the fitness value of the present sparrow, and *f*_*g*_ and *f*_*w*_ are the current global best and worst fitness values, respectively. When *f*_*i*_ > *f*_*g*_, the sparrow is at the edge of the group. When *f*_*i*_=*f*_*g*_, the sparrows that are in the middle of the population are aware of the danger and must move closer to the others.

### 4.2. BP Neural Network

The BP neural network was proposed by Pineda [31] and is widely used. In the BP neural network, the predicted values are generated by linking input layers, hidden layers, and output layers with corresponding weights and thresholds. The weights and thresholds are updated through the gradient descent method by comparing the predicted values and the true response values to minimize the prediction error. The details of the algorithm are presented in Figure 2.

1. Suppose that the input layers are *x*_*i*_={*x*_1_, *x*_2_, ⋯*x*_*i*_, ⋯*x*_*d*_}, hidden layers are *b*_*h*_={*b*_1_, *b*_2_, ⋯*b*_*h*_, ⋯*b*_*q*_}, and output layers are *y*_*j*_={*y*_1_, *y*_2_, ⋯*y*_*j*_, ⋯*y*_*l*_}.
2. Initialize the weights and thresholds within the range (0, 1), where the weights and thresholds linking input and hidden layers are denoted as *w*_*ih*_ and *θ*_*h*_, respectively. The weights and thresholds linking hidden and output layers are denoted as *v*_*hj*_ and *δ*_*j*_, respectively.
3. Calculate the values for hidden layers and output layers by *r*_*h*_=*f*(∑_*i*=1_^*d*^*w*_*ih*_*x*_*i*_ − *θ*_*h*_) and *y*_*j*_=*f*(∑_*j*=1_^*l*^*v*_*hj*_*b*_*h*_ − *δ*_*h*_), respectively.
4. Calculate the overall squared error by $E_{k}=1/2\sum_{j=1}^{l}{\left({\hat{y}}_{j}^{k}-y_{j}^{k}\right)}^{2}$, where ${\hat{y}}_{j}^{k}$ and *y*_*j*_^*k*^ are the predicted value and true value, respectively.
5. Calculate the gradient descents for the output layers and hidden layers, which are given by $g_{j}={\hat{y}}_{j}^{k}\left(1-{\hat{y}}_{j}^{k}\right)\left(y_{j}^{k}-{\hat{y}}_{j}^{k}\right)$ and *e*_*h*_=*b*_*h*_(1 − *b*_*h*_)∑_*j*=1_^*l*^*ω*_*hj*_*g*_*j*_, respectively.
6. Update the corresponding weights and thresholds. In particular, the updated weights for output layers are given by *v*_*hj*_^(*t*+1)^=*v*_*hj*_^(*t*)^+*ηg*_*j*_*b*_*h*_, the updated thresholds for output layers are given by *δ*_*j*_^(*t*+1)^=*δ*_*j*_^(*t*))^ − *ηg*_*j*_, the updated weights for hidden layers are given by *w*__*ih*__^(*t*+1)^=*w*__*ih*__^(*t*)^+*ηe*_*h*_*x*_*i*_, and the updated thresholds for hidden layers are given by *δ*_*h*_^(*t*+1)^=*δ*_*h*_^(*t*)^ − *ηe*_*h*_, where *t* is the number of iterations.
7. During training, if the overall error is smaller than a prespecified value, training is complete. Otherwise, return to step 3 for a new training round until the error is smaller than the requirement or the algorithm reaches the maximum training times.

### 4.3. SSA-BP Neural Network Algorithm

Note that the BP neural network with gradient descent may lead to a local minimum rather than the global minimum. Such drawbacks can be handled by optimizing the initial connection weight and threshold. Therefore, many scholars use intelligent optimization algorithms to select the initial connection weight and threshold value of neural networks, including Genetic Algorithm (GA), Particle Swarm Optimization (PSO), Firefly Algorithm (FA), Grey Wolf Optimizer (GWO), and SSA [32–36]. In this study, SSA was used to optimize the initial connection weight and threshold of the BP neural network, and the optimal connection weight and threshold found by SSA were given to the BP neural network to establish the optimal BP neural network model. The specific process of SSA-BP is shown in Figure 3.

  Step 1: build the BP neural network, determine the BP neural network topology, and initialize the connection weight and threshold.
   Step 2: initialize the parameters of the SSA algorithm, including the initial population size, the maximum evolutionary algebra, the proportion of producers in the population, the proportion of sparrows that are aware of the danger in the population, and the safety threshold.
   Step 3: calculate and sort the fitness values of sparrow individuals to determine the optimal fitness values and the worst fitness values and their corresponding positions.
   Step 4: update the position of the producer according to equation (15).
   Step 5: update the position of the scrounger according to equation (16).
   Step 6: update the position of the sparrows that are aware of the danger according to equation (17).
   Step 7: calculate the fitness value of the new position of the sparrow, compare the updated fitness value with the original optimal value, and update the global optimal information.
   Step 8: verify whether the iteration meets the termination condition. If yes, stop the iteration and record the optimal solution, and go on to step 9; otherwise, return to step 3.
   Step 9: the SSA algorithm's iteration stops, and the global optimal solution generated is used as the initial connection weights and thresholds in the training model of the BP neural network.

## 5. User Experiences with Sports Smart Bracelets

### 5.1. Data Collection

A questionnaire was designed based on the user experience indicator system of the sports smart bracelet built above. The questionnaire consisted of 21 questions, which were composed of the user experience indicator system of the sports smart bracelet built above, and was used to test the real perception level of users to relevant indicators. A seven-point Likert scale was used in the questionnaire obtained at this stage. In this study, 50 users were investigated from May 15th to June 30th, 2021.

### 5.2. Construction of Fuzzy Decision Matrix

The indicator system constructed above is considered to be the factor set of the comprehensive evaluation model, the evaluation data are effectively recovered as the evaluation set of the comprehensive evaluation model, and the membership function transformation method is used to establish the fuzzy membership evaluation matrix corresponding to each indicator element, as shown in Table 3.

### 5.3. Determination of the Weight of Decision Indicators

#### 5.3.1. Analytic Hierarchy Process

Ten experts first made judgments on the importance of each indicator. Based on their opinions, the judgment matrices of first-level and second-level indicators were established. The weight vectors of the first-level indicators and second-level indicators were solved according to equations (3), (4), and (5), as shown in Table 4.

According to equation (6), equation (7), and Table 2, the consistency of the first-level and second-level indicators is checked. Results are shown in Table 5.

As shown in Table 5, the CR value of each factor is less than 0.1, which indicates that all indicators pass the consistency test.

#### 5.3.2. Entropy Weight Method

According to Table 3, the fuzzy synthesis matrix of each second-level indicator under each first-level indicator can be described as follows:

(18) $$\begin{array}{c} T_{1}=\left[\begin{array}{ccccccc} 0 & 0.02 & 0.04 & 0.12 & 0.34 & 0.26 & 0.22\\ 0 & 0.02 & 0.04 & 0.16 & 0.3 & 0.24 & 0.24\\ 0.02 & 0.02 & 0.08 & 0.12 & 0.34 & 0.22 & 0.2 \end{array}\right]\left(0\leq t_{ij}\leq 1\right), \end{array}$$

(19) $$\begin{array}{c} T_{2}=\left[\begin{array}{ccccccc} 0 & 0 & 0.06 & 0.2 & 0.18 & 0.38 & 0.18\\ 0 & 0.04 & 0.06 & 0.18 & 0.22 & 0.3 & 0.2\\ 0 & 0 & 0.06 & 0.18 & 0.2 & 0.36 & 0.2 \end{array}\right]\left(0\leq t_{ij}\leq 1\right), \end{array}$$

(20) $$\begin{array}{c} T_{3}=\left[\begin{array}{ccccccc} 0 & 0 & 0 & 0.2 & 0.24 & 0.34 & 0.22\\ 0 & 0 & 0.04 & 0.16 & 0.26 & 0.28 & 0.26\\ 0 & 0 & 0.04 & 0.22 & 0.24 & 0.32 & 0.18\\ 0 & 0 & 0.02 & 0.14 & 0.32 & 0.24 & 0.28 \end{array}\right]\left(0\leq t_{ij}\leq 1\right), \end{array}$$

(21) $$\begin{array}{c} T_{4}=\left[\begin{array}{ccccccc} 0 & 0 & 0 & 0.12 & 0.34 & 0.3 & 0.24\\ 0 & 0.02 & 0.04 & 0.16 & 0.36 & 0.24 & 0.18\\ 0.02 & 0 & 0.12 & 0.12 & 0.28 & 0.28 & 0.18 \end{array}\right]\left(0\leq t_{ij}\leq 1\right), \end{array}$$

(22) $$\begin{array}{c} T_{5}=\left[\begin{array}{ccccccc} 0 & 0.02 & 0.04 & 0.12 & 0.26 & 0.26 & 0.3\\ 0 & 0 & 0.04 & 0.12 & 0.26 & 0.3 & 0.28\\ 0.02 & 0 & 0.02 & 0.12 & 0.28 & 0.32 & 0.24 \end{array}\right]\left(0\leq t_{ij}\leq 1\right). \end{array}$$

According to equations (18)–(22), the objective weight vector of each evaluation indicator is obtained by the EWM, as shown in Table 6.

#### 5.3.3. Comprehensive Weighting Method to Calculate the Weight of Each Indicator

To avoid the excessive subjectivity of the AHP and the separation from the reality of the EWM, this study uses the comprehensive weighting method to combine the two, and results are shown in Tables 7 and 8.

Table 8 and Figure 4 highlight the importance of each indicator in the 16 evaluation indicators. The movement mode and heart rate detection are the most important indicators for experts and evaluators. These two indicators highlight that the focus of the sports smart bracelet is on human health exercise function and heart rate detection function. The second important result is that device synergy is linked to interactivity; thus, whether the device can deliver data to the user in a timely manner is important for sports smart bracelets. In addition, the sports smart bracelet's body sensing and touch interface is more important than its size, color, shape, and other features of the device, which shows that the user must be an integral part of the sports smart bracelet's interactive features.

### 5.4. Fuzzy Comprehensive Evaluation

According to Tables 3 and 8 and equation (14), a fuzzy comprehensive evaluation calculation for each indicator layer can be obtained:

(23) $$\begin{array}{c} R_{1}=W_{1}{}^{T}\times T_{1}=\left(0.0065,0.02,0.053,0.1294,0.3306,0.2423,0.2182\right),\\ R_{2}=W_{2}{}^{T}\times T_{2}=\left(0,0.0115,0.0601,0.1860,0.2001,0.3490,0.1943\right),\\ R_{3}=W_{3}{}^{T}\times T_{3}=\left(0,0,0.0201,0.1693,0.2792,0.2832,0.2483\right),\\ R_{4}=W_{4}{}^{T}\times T_{4}=\left(0.0032,0.0059,0.0310,0.1318,0.3363,0.2790,0.2126\right),\\ R_{5}=W_{5}{}^{T}\times T_{5}=\left(0.0058,0.0091,0.0342,0.1200,0.2658,0.2876,0.2775\right),\\ T=\left[\begin{array}{ccccccc} 0.0065 & 0.02 & 0.053 & 0.1294 & 0.3306 & 0.2423 & 0.2182\\ 0 & 0.0115 & 0.0601 & 0.186 & 0.2001 & 0.349 & 0.1943\\ 0 & 0 & 0.0201 & 0.1693 & 0.2792 & 0.2832 & 0.2483\\ 0.0032 & 0.0059 & 0.031 & 0.1318 & 0.3363 & 0.279 & 0.2126\\ 0.0058 & 0.0091 & 0.0342 & 0.12 & 0.2658 & 0.2876 & 0.2775 \end{array}\right]\left(0\leq t_{ij}\leq 1\right),\\ L=W^{T}\times T=\left(0.0013,0.0054,0.0328,0.1618,0.2725,0.2907,0.2347\right). \end{array}$$

According to these results, only 3.95% of the users are relatively dissatisfied with the product; 27.25% of users are satisfied with the product; 29.07% of users are satisfied with the product as a whole; and 23.47% of users are very satisfied with the product as a whole.

According to the indicators of each level, 46.05%, 54.33%, 53.15%, 49.16%, and 56.15% of users were satisfied with the appearance characteristics, interactivity, function, material, and product characteristics, respectively. Users' satisfaction with the appearance features and materials of the product is relatively low. Designers must consider these two aspects when developing a product, particularly its appearance.

### 5.5. SSA-BP and BP Neural Network Model Verification

The application of fuzzy comprehensive evaluation to the user evaluation of the sports intelligent wristband can describe the user's satisfaction with the product to some extent, but the weight calculation is complex. To effectively ensure the accuracy of the evaluation results while ensuring fast evaluation results, we use a BP neural network to model each evaluator's score for the sports smart bracelet, predict the comprehensive evaluation score of the sports smart bracelet, and use SSA to optimize the BP neural network. The amount of sample data collected in this study is 50, each sample has 16 variables, and the comprehensive evaluation score Y is calculated as the target variable based on the fuzzy comprehensive evaluation weights obtained above. Some data are shown in Table 9.

#### 5.5.1. Parameter Selection and Performance Indicators

The BP neural network is structured as follows: the number of neurons in the input layer is 16, the number of neurons in the output layer is 1, the maximum number of training iterations is 1000, the minimum error of the training target is 0.00001, and the learning rate is 0.01. According to the empirical formula, the number of neurons in the hidden layer can be calculated as follows: *h*_0_=5 and *h*_max_=14. The SSA initialization parameters are as follows: the initial population size is 30, the maximum number of iterations is 50, producers account for 20% of the population, sparrows that are aware of the danger account for 20% of the population, and the safety threshold is 0.6. To obtain a more intuitive sense of the prediction accuracy of the model, we selected 4 performance indicators to evaluate the model: mean square error (MSE), root mean square error (RMSE), mean absolute error (MAE), and mean absolute percentage error (MAPE) [37]:

(24) $$\begin{array}{c} \text{MSE}=\frac{1}{n}\sum_{i=1}^{n}{\left({\hat{y}}_{i}-y_{i}\right)}^{2},\\ \text{RMSE}=\sqrt{\frac{1}{n}\sum_{i=1}^{n}{\left({\hat{y}}_{i}-y_{i}\right)}^{2}},\\ \text{MAE}=\frac{1}{n}\sum_{i=1}^{n}\left|{\hat{y}}_{i}-y_{i}\right|,\\ \text{MAPE}=\frac{100\%}{n}\sum_{i=1}^{n}\left|\frac{{\hat{y}}_{i}-y_{i}}{y_{i}}\right|, \end{array}$$

where ${\hat{y}}_{i}$ and *y*_*i*_ are the predicted and true values for the *i*th observation, respectively, and *n* is the number of observations.

MSE is used to detect the deviation between the predicted value and the real value of the model. The smaller the MSE is, the better the accuracy of the model is in describing the experimental data. RMSE takes the square root of the MSE to measure the deviation between the observed value and the true value. MAE is the average absolute error, which can describe the real situation of predicted value error with more accuracy. MAPE divides MAE by the true value and then multiplies by percentage, which can describe relative errors with more accuracy.

#### 5.5.2. Determination of the Number of Hidden Layer Neurons

Figure 5 shows that when the number of neurons in the hidden layer is 7, the MSE of the model is minimized; thus, the number of neurons in the hidden layer is set to 7 to train the model.

#### 5.5.3. Comparison of Results

In Figure 6, we found that the predicted value of SSA-BP model is closer to the true value compared with basic BP model, which indicates that the SSA-BP model produces better estimates by integrating the parameter optimization scheme with basic BP model. Furthermore, we compare the performances of different optimization algorithms. To be more specific, in Figure 7, we discover that the SSA-BP model produces smaller error compared to GA-BP and PSO-BP models, which indicates a more accurate estimate.

To further increase the reliability of the prediction results, the MAE, MSE, RMSE, and MAPE of SSA-BP and BP are compared, as shown in Table 10.

In Table 10, SSA-BP generates smaller MAE compared to BP, GA-BP, and PSO-BP models with decreases of 98.02%, 95.97%, and 95.27%, respectively. Similarly, SSA-BP generates smaller MSE than BP, GA-BP, and PSO-BP models with decreases of 99.97%, 99.84%, and 99.81%, respectively. Consistent results can be found in other performance measures like RMSE and MAPE. All results indicate that SSA improves the prediction accuracy of basic BP model and is more effective than other optimization algorithms like GA and PSO.

### 5.6. Discussion

In this study, 16 second-level indicators were selected and divided into 5 first-level indicators. The advantages of the proposed method in this field of study were confirmed through a user experience study of sports smart bracelets. The importance of each index was first judged by 10 experts, and the judgment matrix of the first-level and second-level indices was established based on their opinions. The weight of each evaluation index was calculated by the analytic hierarchy process and the consistency of each evaluation index was tested. Then, the entropy weight method and fuzzy membership evaluation matrix are used to determine the weight of each index. Then, integrating the results using the comprehensive weighted method, we obtain the comprehensive weights which indicates that health-related movement patterns and heart rate detection are shown to be the most important indicators for both experts and users. The second important result is the interaction of equipment coordination, body induction and touch screen, the weight of the above equipment size, color, and shape. Both experts and users attach more importance to the man-machine communication function of sports smart wristband. Thus, the final comprehensive evaluation results indicate that 79.79% of users are satisfied with the product, while the satisfaction of users with the appearance features and materials of the product is relatively low. Designers must consider these two aspects, particularly product appearance, when developing the product. To avoid tedious weight calculation, this study creatively uses the SSA-BP neural network to conduct a comprehensive evaluation of sports smart bracelets. Using the MSE, RMSE, MAE, and MAPE evaluation models, SSA-BP is shown to achieve better results than GA-BP, PSO-BP, and basic BP models.

## 6. Conclusions and Future Work

Facing a series of chronic diseases caused by obesity and overweight, physical exercise is an effective way to prevent these chronic diseases. A high-quality sports smart bracelet can provide convenience for people during physical exercise. How to evaluate a smart sports bracelet quickly and accurately has become a critical problem. In this study, we use fuzzy comprehensive evaluation to evaluate sports smart bracelets. Fuzzy comprehensive evaluation must determine the weight of each indicator, and many scholars have used AHP or EWM for this purpose [38, 39]; however, only AHP is used to determine the weight of each evaluation indicator in this study, which makes it easy to obtain decision results with a certain degree of subjectivity. If the EWM is used to determine the weight of each evaluation indicator, it is easy to become divorced from reality. This study combines the two methods through the comprehensive weighting method and obtains the comprehensive weight of the indicator to perform the comprehensive evaluation of the product, which can help the decision-maker to evaluate a product more scientifically and accurately and provide a basis for decisions when developing new products. In the evaluation of sports smart wristbands, when determining the weight of comprehensive indicators, we found that movement mode and heart rate detection were the most important indicators for both experts and users, followed by device collaboration, motion sensing, and touch interfaces in terms of interaction, indicating that users attach great importance to functionality and interaction. In the final comprehensive evaluation, users' satisfaction with the appearance features and materials of the product is relatively low. Thus, designers must focus on these aspects when developing the product in the future. Second, to avoid cumbersome weight calculations, this study uses the SSA-BP neural network to comprehensively evaluate sports intelligence bracelets. Results show that the SSA optimized BP neural network model achieves good predictions and can effectively ensure the accuracy of evaluation results while ensuring rapid motion evaluation results of intelligent bracelets.

Additionally, this study has certain limitations, and its results should be considered in future research. (1) Using the analytic hierarchy process and entropy weight method and fuzzy comprehensive evaluation method to evaluate single existing products, we plan to consider evaluating the design of multiple auxiliary decision-makers to select the best auxiliary decision-makers for plan optimization. (2) The intelligent optimization algorithm must also initialize relevant parameters. Selecting parameters to reduce model error and improve prediction accuracy when evaluating products should be investigated in more detail. (3) Evaluating existing products is an important step in new product development; thus, in future research, other methods such as ELECTRE III or DEMATEL (Decision-Making Trial and Evaluation Laboratory) could bring valuable solutions [40, 41].

## Figures and Tables

**Figure 1:** Sports smart bracelet user experience indicator system.

**Figure 2:** BP neural network structure.

**Figure 3:** Flow chart of SSA-BP neural network algorithm.

**Figure 4:** Weight of each evaluation indicator of AHP + EWM relative to the overall goal.

**Figure 5:** MSE for different hidden layers.

**Figure 6:** Prediction results of each model.

**Figure 7:** Comparison chart of relative error of each model.

**Table 1:** Recent literature on the comprehensive evaluation methods.

Author	AHP	EWM	FCE	Product evaluation
Zheng et al. [13]	√		√	√
Xia et al. [14]	√		√	√
Chang et al. [15]	√		√	√
Li et al. [16]		√		√
Hayat et al. [17]		√		√
Ma et al. [19]	√	√		
Zhang et al. [18]	√	√	√	

AHP, analytic hierarchy process; EWM, entropy weight method; FCE, fuzzy comprehensive evaluation.

**Table 2:** Random consistency indicators.

Dimension	RI
1	0
2	0
3	0.52
4	0.89
5	1.12
6	1.26
7	1.36
8	1.41
9	1.46
10	1.49
11	1.52
12	1.54
13	1.56
14	1.58
15	1.59
16	1.5943
17	1.6064
18	1.6133
19	1.6207
20	1.6292

**Table 3:** Fuzzy membership evaluation matrix of user experience of sports smart bracelets.

First-level indicators	Second-level indicators	Comment set						
		*P*1	*P*2	*P*3	*P*4	*P*5	*P*6	*P*7
Appearance characteristic S1	Size S11	0	0.02	0.04	0.12	0.34	0.26	0.22
	Color matching S12	0	0.02	0.04	0.16	0.3	0.24	0.24
	Modeling design S13	0.02	0.02	0.08	0.12	0.34	0.22	0.2

Interactive S2	Somatosensory inductive S21	0	0	0	0.2	0.18	0.38	0.18
	Touch interface S22	0	0.4	0.6	0.18	0.22	0.3	0.2
	Device synergy S23	0	0	0.6	0.18	0.2	0.36	0.2

Functional S3	Heart rate detection S31	0	0	0	0.2	0.24	0.34	0.22
	Detection of sleep S32	0	0	0.04	0.16	0.26	0.28	0.26
	Blood oxygen detection S33	0	0	0.04	0.22	0.24	0.32	0.18
	Motor function S34	0	0	0.02	0.14	0.32	0.24	0.28

Material S4	Material softness S41	0	0	0	0.12	0.34	0.3	0.24
	Material breathability S42	0	0.02	0.04	0.16	0.36	0.24	0.18
	Material cleanliness S43	0.02	0	0.12	0.12	0.28	0.28	0.18

Product characteristics S5	Battery endurance S51	0	0.02	0.04	0.12	0.26	0.26	0.3
	Waterproof properties S52	0	0	0.04	0.12	0.26	0.3	0.28
	Charging way S53	0.02	0	0.02	0.12	0.28	0.32	0.24

*Note.P* 1 is “very dissatisfied,” *P* 2 is “dissatisfied,” *P* 3 is “relatively dissatisfied,” *P* 4 is “uncertain,” *P* 5 is “relatively satisfied,” *P* 6 is “satisfied,” and *P* 7 is “very satisfied.”

**Table 4:** Weight of user experience evaluation indicators of sports smart bracelets based on AHP.

Target	First-level indicators	Weights	Second-level indicators	Weights
Sports smart bracelet user experience	S1	0.138	S11	0.444
			S12	0.258
			S13	0.298
	S2	0.244	S21	0.256
			S22	0.364
			S23	0.379
	S3	0.455	S31	0.244
			S32	0.173
			S33	0.139
			S34	0.445
	S4	0.075	S41	0.429
			S42	0.339
			S43	0.232
	S5	0.088	S51	0.486
			S52	0.237
			S53	0.277

**Table 5:** Consistency test.

Level	*λ*_max_	_CI_	_CR_
All	5.07080	0.01770	0.00002
S1	3.00143	0.00071	0.00120
S2	3.01110	0.00550	0.00960
S3	4.00500	0.00170	0.00180
S4	3.00070	0.00036	0.00061
S5	3.00070	0.00033	0.00057

**Table 6:** Weights of evaluation indicators of user experience of sports smart bracelets based on EWM.

Target	First-level indicators	Weights	Second-level indicators	Weights
Sports smart bracelet user experience	S1	0.177	S11	0.332
			S12	0.305
			S13	0.363
	S2	0.169	S21	0.376
			S22	0.259
			S23	0.365
	S3	0.277	S31	0.284
			S32	0.228
			S33	0.229
			S34	0.259
	S4	0.188	S41	0.448
			S42	0.308
			S43	0.244
	S5	0.188	S51	0.304
			S52	0.356
			S53	0.339

**Table 7:** Weight of evaluation indicator of user experience of sports smart bracelets based on AHP and EWM.

Target	First-level indicators	Weights	Second-level indicators	Weights
Sports smart bracelet user experience	S1	0.11	S11	0.441
			S12	0.235
			S13	0.324
	S2	0.185	S21	0.293
			S22	0.287
			S23	0.421
	S3	0.567	S31	0.271
			S32	0.154
			S33	0.124
			S34	0.451
	S4	0.063	S41	0.544
			S42	0.296
			S43	0.16
	S5	0.074	S51	0.453
			S52	0.259
			S53	0.288

**Table 8:** Weight of each evaluation indicator relative to the overall goal based on multiple methods.

Indicators	AHP	EWM	AHP + EWM
S11	0.061	0.06	0.057
S12	0.036	0.055	0.031
S13	0.041	0.066	0.042
S21	0.062	0.065	0.063
S22	0.089	0.045	0.063
S23	0.092	0.063	0.091
S31	0.111	0.081	0.141
S32	0.079	0.055	0.068
S33	0.063	0.05	0.049
S34	0.202	0.073	0.23
S41	0.032	0.086	0.043
S42	0.025	0.059	0.023
S43	0.017	0.047	0.012
S51	0.043	0.059	0.04
S52	0.021	0.069	0.023
S53	0.024	0.065	0.024

**Table 9:** Evaluation of user experience of sports smart bracelets (part).

Number	S11	S12	S13	…	S51	S52	S53	Y
…	…	…	…	…	…	…	…	…
12	5	5	5	…	5	5	5	5
13	3	3	3	…	5	5	5	4.306
14	5	3	3	…	5	3	5	4.74
15	5	5	5	…	5	5	7	5.067
16	7	2	2	…	7	7	7	5.699
17	6	6	6	…	7	7	6	6.215
18	6	6	6	…	6	6	6	6
…	…	…	…	…	…	…	…	…

**Table 10:** Performance comparison of each model under different evaluation indicators.

Model	MAE	MSE	RMSE	MAPE (%)
BP	0.23657	0.10768	0.32814	4.508
SSA-BP	0.0046943	3.1148*e* − 05	0.0055811	0.091783
GA-BP	0.11659	0.019531	0.13975	2.2018
PSO-BP	0.09928	0.016239	0.12743	1.9276

## Data Availability

The data used to support the findings of this study are available from the corresponding author upon request.
